# The Association of Polymorphisms in *Nrf2* and Genes Involved in Redox Homeostasis in the Development and Progression of Clear Cell Renal Cell Carcinoma

**DOI:** 10.1155/2021/6617969

**Published:** 2021-04-17

**Authors:** Smiljana Mihailovic, Vesna Coric, Tanja Radic, Ana Savic Radojevic, Marija Matic, Dejan Dragicevic, Milica Djokic, Vladimir Vasic, Zoran Dzamic, Tatjana Simic, Jovan Hadzi-Djokic, Marija Pljesa Ercegovac

**Affiliations:** ^1^The Obstetrics and Gynaecology Clinic Narodni Front, 11000, Serbia; ^2^Institute of Medical and Clinical Biochemistry, 11000, Serbia; ^3^Faculty of Medicine, University of Belgrade, 11000, Serbia; ^4^Institute of Mental Health Belgrade, 11000, Serbia; ^5^Clinic of Urology, Clinical Center of Serbia, 11000, Serbia; ^6^Institute for Oncology and Radiology of Serbia, 11000, Serbia; ^7^Department of Urology, University Medical Center Zvezdara, 11000, Serbia; ^8^Serbian Academy of Sciences and Arts, 11000, Serbia

## Abstract

Deleterious effects of SNPs found in genes encoding transcriptional factors, as well as antioxidant and detoxification enzymes, are disputable; however, their functional significance seems to modify the risk for clear cell renal cell carcinoma (ccRCC) development and progression. We investigated the effect of specific *Nrf2*, *SOD2*, *GPX1* gene variants and *GSTP1ABCD* haplotype on ccRCC risk and prognosis and evaluated the association between GSTP1 and regulatory (JNK1/2) and executor (caspase-3) apoptotic molecule expression in ccRCC tissue samples and the presence of GSTP1 : JNK1/2 protein : protein interactions. Genotyping was performed in 223 ccRCC patients and 336 matched controls by PCR-CTTP and qPCR. Protein expression was analyzed using immunoblot, while the existence of GSTP1 : JNK1 protein : protein interactions was investigated by immunoprecipitation experiments. An increased risk of ccRCC development was found among carriers of variant genotypes of both *SOD2* rs4880 and *GSTP1* rs1695 polymorphisms. *Nrf2* rs6721961 genetic polymorphism in combination with both rs4880 and rs1695 showed higher ccRCC risk as well. Haplotype analysis revealed significant risk of ccRCC development in carriers of the *GSTP1C* haplotype. Furthermore, GSTP1 variant forms seem to affect the overall survival in ccRCC patients, and the proposed molecular mechanism underlying the GSTP1 prognostic role might be the presence of GSTP1 : JNK1/2 protein : protein interactions.

## 1. Introduction

Cellular redox homeostasis is maintained by constant metabolic fluxes and redox feedback consisting of electrophilic molecules produced by all kinds of stressors that activate diverse mechanisms aimed at reestablishing nucleophilic environment [1]. Disturbance of this fine balance between reactive oxygen species (ROS) production and their disintegration leads to oxidative stress and cellular damage on multiple levels [2]. In order to adapt, a phenotypic switch has to take place [1]. Cells that have a high proliferation rate, such as cancer cells, demand constant energy production to maintain biosynthesis of macromolecules. In order to adapt and support their basic needs, both intrinsic and extrinsic molecular mechanisms are involved in modifying cellular metabolism [3]. While constantly rapidly proliferating, cancer cells are, at the same time, exposed to increased ROS levels, which further upregulate antioxidant systems and create environment in which they are able to develop new redox balance and resistance to oxidative damage [3].

Clear cell renal cell carcinoma (ccRCC) remains one of the most frequent and the most aggressive adult renal malignancies, accounting for up to 90% of all kidney tumors [4, 5]. Since alterations in metabolism are among ccRCC hallmarks, it has been suggested that besides histological classification of RCC, certain molecular subtypes should also be identified [6, 7]. Precise classification is of utmost importance, since it might reveal types with more or less aggressive clinical features and therefore point out which patients should be more closely monitored and followed [8].

Clear cell RCC belongs to types of carcinomas associated with Keap1/Nrf2 (Kelch-like ECH-associated protein 1/nuclear factor (erythroid-derived 2)-like2) pathway alterations [8]. Namely, when cellular levels of reactive oxygen species and electrophiles are increased, specific adaptive cytoprotective response is activated, including changes in the Keap1/Nrf2 pathway [9, 10]. Induced allosteric changes in Keap1 lead to decreased proteasomal degradation of the transcriptional factor Nrf2 [10]. Once accumulated, Nrf2 enters the cell nucleus and binds to antioxidant response element (ARE) DNA sequences of Nrf2 target genes, further causing intensified transcription of numerous enzymes, including detoxifying enzymes, metabolic enzymes, and stress response proteins [8, 10, 11]. Although at first perceived as an anticancer molecule, some authors emphasize the role of Nrf2 in cancer cell survival and even suggest that it should be regarded as a possible target for future anticancer therapeutic approaches [9, 12, 13].

Among various enzymes encoded by Nrf2 target genes and regulated by their binding to AREs are glutathione S-transferases (GST). They represent a family of multifunctional enzymes involved in a number of catalytic and noncatalytic processes, still traditionally recognized as phase II cellular detoxification system enzymes [3, 14]. The liver, lung, and kidneys, as organs with intense metabolic activity, are known to have high expression of cytosolic GSTs, especially the pi (GSTP) form, whose gene activation is regulated by Nrf2 [14, 15]. GSTP1 also possesses binding activity toward macromolecules, as well as small molecules, and displays ability to participate in a large signal transduction pathway [14, 16]. Specifically, GSTP1 acts as a negative regulator of kinase-dependent apoptotic signaling pathways by forming protein : protein complexes with regulatory mitogen-activated kinases such as JNK1 (c-Jun NH2-terminal kinase) [14, 17]. The particular GSTP1 : JNK1 interaction has gained attention as the new, functional link between the upregulated GSTP1 and malignant phenotype [3]. Additionally, GSTP1 has a potential to form a GSTP1/Nrf2 protein complex, suggesting a possibility that GSTP1 protein might help Nrf2 stabilization and its further actions [18]. When considering its role in cancer metabolism, in addition to detoxification of potential cancerogenic substances, GSTP1 is capable of increasing drug efflux from the cell thus contributing to chemoresistance [19].

Since cancer cells are energy-dependent, metabolic reprogramming is the basis of their sustenance [7]. In order to keep up with high energy demands and to defend themselves from many reactive molecules, tumor cells rely on enzymes that enable both processes [20, 21]. There are three isoenzymes of SOD, a major antioxidant enzyme [22]. In the reaction catalyzed by mitochondrial SOD2, H_2_O_2_, a well-known molecule with novel functions in cell proliferation, differentiation, and migration, is being produced. In addition to acting as a signaling molecule, H_2_O_2_ facilitates activation of AMP-activated kinase and promotes glycolysis which is a key change for cancer cells [20, 22]. Therefore, by controlling the H_2_O_2_ production, SOD2 plays an important role in numerous pathways.

And while SOD2 leads to H_2_O_2_ synthesis, another key antioxidant enzyme, glutathione peroxidase (GPX), leads to its further reduction and production of a neutral water molecule [23]. Eight members comprise the GPX family [24]. By helping cancer cells eliminate potentially harmful hydrogen peroxide, the role of GPX1 as the most abundant GPX form might be contradictory [25]. Namely, its increased activity protects normal cells from oxidative damage, while this could be helpful for cancer cells to escape ROS as well [25].

Both the Nrf2 gene and genes encoding GSTP1, SOD2, and GPX1 have functional polymorphisms, which either change the level of expression of specific protein or affect the activity of synthesized proteins. The widely analyzed *Nrf2* SNP polymorphism rs6721961 involves substitution of C to A, positioned at -617 of the proximal promoter [26]. Definite consequent functional changes are still unsolved, and it is discussed whether higher or lower transcriptional activity is associated with a variant-type genotype (-617AA) [27]. However, since this SNP is located in the ARE-like motif of the gene, importance for self-induction of the *Nrf2* is being emphasized throughout the literature [26, 28, 29]. In the case of *GSTP1* gene polymorphisms, two most commonly occurring SNPs are rs1695 and rs1138272 [30]. Substitution of A313G in the case of rs1695 causes change of isoleucine with valine at position 105 (Ile105Val) [31]. This *Val* allele variant represents a more potent c-Jun N-terminal kinase 1 (JNK1) inhibitor and has a stronger antiapoptotic effect [32]. The presence of T instead of C at position 341 results in coding of protein with valine instead of alanine (rs1138272, Ala114Val) [33]. It is assumed that the 341T variant of GSTP might have decreased activity or modified substrate specificity [34]. The haplotype *GSTP1ABCD* represents a combination of these two polymorphisms. When it comes to *SOD2* polymorphism, rs4880 corresponds to substitution of C>T in exon 2 leading to change from alanine to valine at position 16 [35]. Since there is a channel within the inner mitochondrial membrane that cannot import the Val16 variant of SOD2 as efficiently as Ala16, the Val16 variant remains trapped and later degraded by the proteasome [35]. The mostly studied SNP in the case of the *GPX1* gene is rs1050450 (Pro200Leu). Due to change of proline with leucine, secondary and tertiary structures of GPX1 are altered, leading to conformational change of the enzyme as a whole [36]. Proline is basically essential, because of its unsubstituted amino group on the *α* carbon atom which enables formation of a specific kink; therefore, when absent, the whole structure is modified [36].

Considering the potential functional significance of polymorphisms in genes encoding the Nrf2 transcriptional factor, as well as antioxidant SOD2, GPX1, and detoxification GSTP1 enzymes in both the onset and prognosis of clear cell RCC, the aim of this study was to evaluate the effect of specific *Nrf2*, *SOD2*, and *GPX1* gene variants and *GSTP1ABCD* haplotype on the risk, development, and postoperative prognosis in patients with ccRCC. Furthermore, the aim was to evaluate the association between GSTP1 expression and expression of regulatory (JNK1/2) and executor (caspase-3) apoptotic molecules in human ccRCC tissue samples, as well as the presence of GSTP1 : JNK1/2 protein : protein interactions.

## 2. Materials and Methods

### 2.1. Participants

The case-control study included 223 patients with histologically confirmed clear cell renal cell carcinoma treated and followed at the Clinic of Urology of Clinical Center of Serbia, Belgrade. Incident cases were recruited at the time of diagnosis which included the presence of malignantly enhanced lesions detected by imaging techniques and confirmed by histological diagnosis. Obtained blood and tissue samples were assessed within the Biobank formed in the Laboratory for Functional Genetics and Proteomics at the Institute of Medical and Clinical Biochemistry of the Faculty of Medicine, University of Belgrade. The enrolled 336 controls were gender- and age-matched cancer-free subjects. These individuals with no previous history of cancer had undergone surgery for benign conditions at the same clinical center, unrelated to both nonmalignant and malignant urological conditions. Participants gave their informed consent for inclusion in the study. The study was conducted in accordance with the Declaration of Helsinki, and the protocol was approved by the Ethics Committee of the Faculty of Medicine, University of Belgrade (no. 29/X-3). Both cases and controls were interviewed using a standard epidemiological questionnaire in order to gain information about risk factors for ccRCC development. Smokers were defined as subjects who had a period of at least 60 days of consuming cigarettes prior to inclusion in the study. Pack-years was calculated by the formula pack‐years = (cigarettes/day ÷ 20) × years of smoking. Overall survival was defined as time from nephrectomy to the date of death or last follow-up (November 2018).

### 2.2. DNA Isolation

Genomic DNA was isolated from 200 *μ*l of the whole blood sample or from 25 mg of distant nontumor kidney tissue samples, using a QIAamp DNA mini kit (Qiagen, Chatsworth, CA, USA). Isolated DNA was stored at -20°C. The concentration, as well as purity of isolated DNA, was measured by spectrophotometry at 230, 260, 280, and 320 nm on GeneQuant pro (Biochrom, Cambridge, England).

### 2.3. Analysis of Examined Genotypes

The polymorphism rs6721961 for *Nrf2* was examined by the PCR-CTTP (polymerase chain reaction with confronting two-pair primers) method according to Shimoyama et al. [37]. Products of amplification were divided by electrophoresis with 2% agarose gel. Visualization of PCR products was enabled with SYBR® Safe DNA Gel Stain (Invitrogen Corporation, Carlsbad, California, USA) on a UV ChemiDoc camera (Bio-Rad, Hercules, California, USA). A lane containing 282 and 113 bp was considered a C/C genotype; a lane with 282, 205, and 113 bp, a heterozygous genotype; and a lane with 282 and 205 bp, a A/A genotype.

Genotyping of *GSTP1* (rs1695 and rs1138272), *SOD2* (rs4880), and *GPX1* (rs1050450) was done by applying quantitative polymerase chain reaction (qPCR) on Mastercycler ep realplex (Eppendorf, Hamburg, Germany) using appropriate assays of Applied Biosystems TaqMan Drug Metabolism Genotyping (Life Technologies, Applied Biosystems, Carlsbad, CA, USA). Assays C_3237198_20 in the case of *GSTP1* rs1695, C_1049615_20 for *GSTP1* rs1138272, and C_8709053_10 were used for *SOD2*. For the *GPX1* rs1050450 polymorphism, a custom-designed assay with sequences 5′ VIC-ACAGCTGGGCCCTT-MGB-3′ and 5′ FAM-ACAGCTGAGCCCTT-MGB-3′ was used.

### 2.4. Immunoblot Analysis

Cytosols were obtained from ccRCC tumor (*n* = 20) and respective nontumor kidney tissue samples. A pool of nontumor kidney tissue was made by mixing the equal parts of six different samples. 50 *μ*g of total protein per sample was subjected to immunoblot analysis of JNK1/2, GSTP1, and cleaved caspase-3 expression [38, 39]. Membranes were blocked overnight and treated with primary antibodies against JNK1/2 (Sigma-Aldrich, St. Louis, Missouri, USA), GSTP1 (Abcam, Cambridge, UK), cleaved caspase-3 (Cell Signaling, Danvers, Massachusetts, USA), and housekeeping protein *β*-actin (Sigma-Aldrich, St. Louis, Missouri, USA). Afterwards, membranes were incubated with appropriate secondary antibodies, treated with a chemiluminescence detection substrate (Invitrogen Corporation, Carlsbad, CA, USA), and exposed to X-ray films (Amersham Hyperfilm ECL, GE Healthcare, Buckinghamshire, England). Densitometry analysis was performed using ImageJ (National Institutes of Health, Bethesda, USA). In order to obtain relative quantitation, the results were normalized using *β*-actin housekeeping protein.

In order to investigate the presence of GSTP1 : JNK1 protein : protein interactions in tumor ccRCC samples, immunoprecipitation experiments were performed using Catch and Release® v2.0 High Throughput (HT) Immunoprecipitation Assay Kit-96 well (Upstate Biotech Inc. for Merck Millipore, Darmstadt, Germany) according to the manufacturer's instructions. Namely, a 96-well filter plate was used for a precoating procedure with provided 20% *w*/*v* slurry resign and Affinity Ligand. Selected cytosols, containing 1 *μ*g/*μ*l of total cell proteins, previously quantified by using the Bicinchoninic Acid Protein Assay Kit (BCA-1, Sigma-Aldrich, St. Louis, Missouri, USA) were incubated with 2 *μ*g of the primary antibody against GSTP1 (Cell Signaling, Danvers, Massachusetts, USA), followed by several washing steps. Finally, samples were resuspended in 30 *μ*l of 2x Laemmli buffer (Bio-Rad, Hercules, CA, USA), denatured at 90°C for five minutes, and collected by centrifugation at 1500 rpm for one minute. Supernatant fraction was further subjected to SDS-PAGE and Western blot analysis according to the previously described protocols.

### 2.5. Statistical Analysis

Calculations for this investigation were performed using the SPSS software version 17.0 (Chicago, IL, USA). Continuous variables were expressed as mean ± standard deviation (SD) or median (minimum–maximum). Frequency (*n*, %) counts were used for categorical variables. Distribution of different variables was tested by using the Kolmogorov-Smirnov test. For each examined polymorphism, the Hardy-Weinberg equilibrium was tested. The risk each genetic variant carries for ccRCC development was computed by odds ratios (OR) and 95% confidence intervals (CI) by logistic regression analysis. OR was adjusted for age, gender, and variables indicating recognized risk factors for ccRCC as potential confounders. Survival analysis was performed using the Kaplan-Meier method to estimate the cumulative survival probability. The log-rank test was performed for the assessment of differences in survival according to the different categories of variables. The association between GSTP1 and cleaved caspase-3 expression was analyzed using Spearman's coefficient of linear correlation.

## 3. Results and Discussion

### 3.1. Analysis of Genotypes

The analyzed sample included a total number of 223 ccRCC patients and 336 age- and gender-matched controls with the same geographic origin. The main demographic and clinical features of patients and controls are summarized in Table 1.

As presented, recognized risk factors for ccRCC, history of obesity, hypertension, and smoking status, were evaluated. While no significant difference among groups was found regarding obesity and smoking status, more than 50% of patients were presenting hypertension in comparison with 35% hypertensive controls. Additionally, subjects who had history of hypertension exhibited 2.45-fold increased risk for ccRCC development compared to normotensive subjects (95%CI = 1.375-4.435, *p* < 0.05). Grade II, according to the Fuhrman grading system, was the most prevalent among enrolled cases (106 patients—55%). When staged according to the TNM system, we found pT1 and pT3 to be the most numerous stages (93 pT1 cases and 87 pT3 cases).

The distribution of specific genotypes among ccRCC patients and controls is shown in Table 2.

No significant ccRCC risk was revealed for subjects carrying the C/A and A/A *Nrf2* genotype in comparison with carriers of the C/C genotype (OR = 0.692, 95%CI = 0.370–1.295, *p* = 0.250). On the contrary, the risk for ccRCC development was highly increased in individuals with at least one *SOD2* Val allele or precisely Ala/Val and Val/Val *SOD2* genotypes (OR = 4.521, 95%CI = 2.167–9.432, *p* < 0.001). Regarding *GPX1* polymorphism, the risk for ccRCC development was reduced in subjects carrying Pro/Leu and Leu/Leu genotypes when compared to individuals with the Pro/Pro genotype (OR = 0.567, 95%CI = 0.323–0.994, *p* = 0.048). *GSTP1* polymorphisms rs1695 and rs1138272 were studied individually and in combination, as well as the *GSTP1ABCD* haplotype. As presented, subjects with the Ile/Val and Val/Val rs1695 genotype combined with the Ala/Ala rs1138272 genotype had more than 3-fold increased risk for developing clear cell renal cell carcinoma in comparison with carriers of referent genotypes for both polymorphisms (OR = 3.250, 95%CI = 1.668–6.331, *p* = 0.001).

As a part of an immensely complex redox homeostasis maintenance system, the examined enzymes and their genetic polymorphisms were assessed in combination (Table 3). When observed altogether, subjects with the C/C *Nrf2* genotype who were, at the same time, carrying the Ala/Val or Val/Val *SOD2* genotype, exhibited three-fold increased ccRCC risk (OR 3.234, 95%CI = 1.436–7.280, *p* = 0.005), while subjects with C/A or A/A *Nrf2* in combination with the Ala/Val or Val/Val *SOD2* genotype had 2.9-fold increased risk for ccRCC development (OR = 2.918, 95%CI = 1.131–7.532, *p* = 0.027). Almost equally higher risk was found among carriers of combined C/C *Nrf2* and Ile/Val or Val/Val *GSTP1* rs1695 genotypes (OR = 3.211, 95% CI 1.516–6.814, *p* = 0.002). Logistic regression showed no substantial risk when *Nrf2* genotypes were analyzed in combination with *GPX1* and *GSTP1* rs1138272 genotypes.

The increased ccRCC risk was the most pronounced when *SOD2* and either *GSTP1* rs1695 or rs1138272 polymorphisms were examined. Ala/Val and Val/Val *SOD2* genotypes in combination with Ile/Val and Val/Val rs1695 genotypes were associated with almost 20-fold increased risk (OR = 19.724, 95%CI = 4.267–91.165, *p* < 0.001), while 4-fold increased risk for ccRCC development was observed when in combination with the Ala/Ala *GSTP1* rs1138272 genotype (OR = 4.374, 95%CI = 2.012–9.508, *p* < 0.001). Finally, the presence of the *GPX1* Pro/Pro genotype combined with either the Ala/Val or Val/Val *SOD2* genotype and Ile/Val or Val/Val *GSTP1* rs1695 genotype leads to significantly higher risk for this cancer (OR = 3.653, 95%CI = 1.148–11.630, *p* = 0.028 and OR = 5.476, 95%CI = 2.127–14.102, *p* < 0.001, respectively).

In the next step, haplotype analysis of *GSTP1* rs1695 and rs1138272 polymorphisms was performed and is presented in Table 4. The *GSTP1A* genotype represents a combination of A313 and C114, meaning that the enzyme has isoleucine at position 105 and alanine at 114. The genotype with G313 and C114 or valine at 105 and alanine at 114 is *GSTP1B*. The presence of G313 and T114 or valine at both 105 and 114 represents *GSTP1C*, while the form consisting of isoleucine at position 105 and valine at 114 (A313 and T114) is *GSTP1D* [40]. The haplotype composed of wild-type alleles ∗A and ∗C was the most frequent among ccRCC patients (56%) and controls (64%). Regarding the effect of the GSTP1ABCD haplotype on ccRCC susceptibility, the haplotype consisting of variant alleles of both polymorphisms ∗G and ∗T was associated with 3.5-fold increased risk (OR = 3.50, 95%CI = 1.49–8.22, *p* = 0.004).

### 3.2. Follow-Up Analysis

Of 223 ccRCC cases, follow-up data were acquired for 215 (96%) patients in a period from 2005 to 2018. There were a total number of 80 deaths (37%) and 135 survivals during the mean follow-up period of 67.31 ± 37.68 months (ranging from 1 to 161 months).  Table 5 presents Nrf2, SOD2, GPX1, and GSTP1 genotype distribution among living and deceased ccRCC patients.

Statistically significant difference in frequencies was observed among carriers of Pro/Leu and Leu/Leu genotypes of the examined *GPX1* polymorphism (*p* = 0.024). Regarding the *GSTP1ABCD* haplotype, statistically significant difference in frequencies was observed between carriers of at least one variant allele and carriers of a referent genotype of both *GSTP1* polymorphisms (Table 5).

Table 6 represents the analysis of different examined genotypes as potential predictors for overall mortality. The analysis was performed in two models, based on different adjustments. Although without reaching statistical significance, the *GSTP1*-*variant* genotype consisting of at least one Val105 allele in the case of rs1695, in combination with at least one Val114 allele in the case of rs1138272, expressed the highest hazard ratio in ccRCC patients (model 1 HR = 1.627, 95%CI = 0.664–3.986, *p* = 0.287; model 2 HR = 3.897, 95%CI = 0.681–22.304, *p* = 0.126). On the other hand, none of the other investigated genotypes showed any predicting potential in terms of ccRCC overall mortality.

The Kaplan-Meier survival curves for overall mortality according to *Nrf2*, *GSTP1*, *SOD2*, and *GPX1* genes in ccRCC patients are presented in Figure 1. This analysis for overall survival did not show significantly shorter time of survival in patients carrying a specific *Nrf2*, *SOD2*, or *GPX1* genotype (*p* > 0.05, Figures 1(a), 1(c), and 1(d)). However, patients who were carrying any of variant *GSTP1* genotypes were recognized as patients with shorter overall survival (log-rank *p* = 0.038) (Figure 1(b)).

### 3.3. Analysis of Protein Expression

Since GSTP1 protein may negatively regulate JNK and therefore affect the apoptotic activity, especially within tumor tissue, we analyzed the GSTP1 protein expression both in a pool of nontumor kidney tissue samples and in ccRCC tissue samples, however independently of the *GSTP1* genotype. Moreover, the potential presence of GSTP1 : JNK1/2 complexes was assessed in specimens of tumor tissue obtained from 20 patients with ccRCC. Despite gradual increase in the expression across tumor grades (G1-G3), significant difference was not observed neither for GSTP1 protein levels in ccRCC tissue samples alone (Figure 2, *p* > 0.05) nor between the nontumor kidney tissue pool and ccRCC tissue samples (*p* > 0.05).

Although the JNK1/2 expressed was evidently higher in the nontumor kidney tissue pool in comparison with ccRCC tissue samples (Figure 3), the obtained results were not statistically significant (*p* > 0.05).

Still, the expression of executor cleaved caspase-3 gradually decreased across tumor grade (G1-G3), reaching the statistical significance only in G3, when compared to the pool of nontumor kidney tissue samples (Figure 4, *p* < 0.05).

However, a weak positive correlation (correlation coefficient, *r* < 0.3) was found only between GSTP1 and cleaved caspase-3 expression (*r* = 0.024, *p* = 0.999).

In order to investigate the presence of GSTP1 : JNK1 protein : protein interactions, tumor tissue samples were divided into three groups, according to the tumor's grade. Although the effect of *GSTP1* polymorphic expression was not assessed, the analyzed samples comprised all three GSTP genotypes. Namely, the *GSTP1 IleIle* genotype was present in 30%, *GSTP1 IleVal* in 40%, and *GSTP1 ValVal* in 30% samples. Protein immunoprecipitation, followed by Western blot analysis, showed the presence of JNK1/2/GSTP1 complexes in all assessed ccRCC samples (Figure 5).

## 4. Discussion

In recent years, attention has been raised toward genetic variants, often referred to as “quantitative trait loci” that could contribute to a small, but significant, risk not only for the development but also for the progression of complex disorder such as cancer [41]. Deleterious effects of SNP polymorphisms found in genes encoding transcriptional factors, as well as antioxidant and detoxification enzymes, are still disputable; however, their functional significance might seem to modify the risk for RCC development. Moreover, there is a growing body of evidence that glutathione transferases may participate in tumor progression and affect patients' survival by regulating a number of cellular processes via protein : protein interactions as endogenous negative regulators of protein kinases [16, 17, 42–45].

In this study, we examined the role of genetic polymorphisms of the transcriptional factor Nrf2 and genes coding SOD2 and GPX1, as well as GSTP1, in ccRCC development. We noticed an increased risk of ccRCC development among carriers of variant genotypes of both *SOD2* rs4880 and *GSTP1* rs1695 polymorphisms. *Nrf2* rs6721961 genetic polymorphism in combination with both rs4880 and rs1695 showed higher risk for this type of tumor as well. Since two examined SNPs of *GSTP1*, rs1695 and rs1138272, are close in their position, haplotype analysis was performed. It revealed that significant risk of ccRCC development is associated with a genotype consisting of variant forms of both polymorphisms, while the molecular mechanism underlying the role of GSTP1 forms in RCC progression might be explained by the presence of GSTP1 : JNK1/2 protein : protein interactions.

It has been shown that Nrf2 deficiency decreases the ability of tissue to properly react to exposure to oxidative and electrophilic stressors [46]. The importance of SNP rs6721961 for further Nrf2 activity has been shown, since this polymorphism is positioned in the middle of the ARE motif and affects the binding of Nrf2 to the ARE. Homozygous *A/A* subjects exhibit lower level of Nrf2 mRNA which further leads to lower protein activity [47]. Suzuki et al. demonstrated that smokers—carriers of the *A/ANrf2* genotype—had increased risk of lung cancer development [47], while at the same time, Okano et al. even suggested that this polymorphism should be considered a prognostic biomarker for assessing prognosis in lung adenocarcinoma patients [29]. What is more, women carrying this specific genotype have higher risk for breast cancer development and decreased protein expression in cancer tissue [48].

There are no studies of whether the *Nrf2*-617C/A polymorphism has impact on RCC development. When it comes to tumors of the urinary tract, Reszka et al. found no association between SNP rs6721961 and risk for urinary bladder cancer [27]. Similarly, our results did not show any significant difference in frequencies of different genotypes among ccRCC patients and corresponding controls. Still, in already developed renal cell carcinoma, higher expression of Nrf2 protein in carriers of the *C/C* genotype seems to point out the patients with poor prognosis and shorter overall survival [49]. Furthermore, when the expression of Nrf2 is elevated, RCC metastasis has inadequate and unsatisfying response to therapy which leads to unfavorable outcome [50]. According to our follow-up analysis, patients with the *C/C* genotype did have shorter overall survival compared to *C/A* and *A/A* carriers, although it was not statistically significant.

Many genes targeted by Nrf2 encode enzymes essential in antioxidative stress response which enables cellular adaptation to new conditions [47]. Glutathione S-transferases as enzymes regulated by Nrf2 activity take part in defense against stressors [51]. Although meta-analysis did not find association between *GSTP1* rs1695 polymorphism and RCC development [31, 52], the results of our previous studies on RCC patients indeed demonstrated a significantly increased risk for cancer development in patients carrying the *GSTP1*-*variant* (*Ile/Val+Val/Val*) genotype [16], which was in line with the results obtained on the subpopulation of ccRCC patients [53]. In addition to rs1695, in this study, we analyzed rs1138272 SNP as well. There was significant difference in distribution of the rs1695 genotype among patients and controls, but no association between ccRCC and rs1138272. Four haplotypes involving these two polymorphisms have been defined. Maniglia et al. found haplotypes *GSTP1A* and *GSTP1D* having higher frequency among cases of head and neck squamous cell carcinoma than among controls [54]. Since the overall functions of GSTs also include the regulation of cell signaling, the *GSTP1C* haplotype has been considered a better c-Jun N-terminal kinase 1 inhibitor than the reference *GSTP1A* haplotype [32]. In line with these results, our study showed higher risk for ccRCC for carriers of the *GSTP1C* haplotype.

Based on the established role of the GSTPi class in inhibition of JNK1 and its antiapoptotic effect [17, 45], we assessed the expression of GSTP1 and expression of regulatory (JNK1/2) and executor (caspase-3) apoptotic molecules in human ccRCC tissue samples, as well as the presence GSTP1 : JNK1/2 protein : protein interactions, however irrespective of the *GSTP1* genotype. At first, we noticed gradual increase in the GSTP1 protein across tumor grades, although without significant difference. Secondly, our results showed lower level of JNK1/2 expressed in tumor tissue in comparison with nontumor kidney tissue. Furthermore, the expression of cleaved caspase-3, one of the key executory enzymes leading to apoptosis, was statistically significantly decreased in grade 3 when compared to expression in nontumor tissue. In addition, we found a weak, yet positive, correlation between GSTP1 and cleaved caspase-3 expression. Finally, by analyzing ccRCC tissue homogenates, we found GSTP1 : JNK1/2 complexes in all assessed samples. The particular interaction has been found in human leukemia, hepatic carcinoma, bladder cancer, and neuroblastoma cells [55]. Presumably, tumors with upregulated GSTP1, such as RCC, could have their kinase-dependent apoptotic signaling pathways suppressed, owning to negative regulation of JNK1. Thévenin et al. showed that protein produced in carriers of the Val105 and Val114 genotype acts as a better JNK inhibitor [32]. Indeed, our results have shown that carriers of *GSTP1-variant*-type genotypes—(*Ile/Val+Val/Val*) (*Ala/Val+Val/Val*)—exhibited poorer survival. It is important to note that the GSTP-JNK interaction is shown to be redox-dependent with possible formation of oligomeric forms of GSTP and other thiol-containing proteins, such as Prdx both 1 and 6 [56, 57]. Since Prdx6 seems to be responsible for substantial inhibition of GSTP1 heterodimerization, independently of allelic variations, while Prdx1, once released from the GSTP-JNK complex, maintains its peroxidase activity, it seems plausible that genetic variations in Prdx, both 1 and 6, might play a critical role in this context [57].

Another enzyme influenced by Nrf2 is manganese superoxide dismutase. Involvement of polymorphism rs4880 in cancer susceptibility has been extensively investigated. Comprehensive meta-analysis by Wang et al. showed *SOD2* rs4880 polymorphism to be connected with lung cancer [58]. Various meta-analyses found no association between this SNP and urinary bladder or breast cancer risk [21, 59]. Those studies that actually reported increased risk for breast cancer usually reported the Ala/Ala genotype to be the most frequent, although the carriers of the Val16 variant are expected to be at greater cancer risk [60]. Similarly, some authors found aggressive forms of prostate cancer to be associated with the *Ala/Ala* genotype [61]. Atilgan et al. found that risk for development of any kind of histologic subtypes of renal cell carcinoma is increased with *Ala/Val* and *Ala/Ala* genotypes [35]. In our study, when only clear cell carcinoma was observed, carriers of *Ala/Val* and *Val/Val* genotypes were exposed to significantly greater risk. When analyzed in combination with *Nrf2*, *GPX1*, and both rs1695 and rs1138272 *GSTP1* SNPs, significant risk was also noted. In addition, according to our results, overall survival was shorter among patients with *Ala/Val* and *Val/Val* genotypes still without statistical significance. It is suggested that the Val16 variant of SOD2 comprises parts of *β*-sheet structure and therefore is inefficiently transported into the mitochondrial cytosol which diminishes its function and further leads to inadequate superoxide anion neutralization [62]. However, Dasgupta et al. found that excessive H_2_O_2_ production leads to reduced sensitivity to tumor necrosis factor-*α*-mediated apoptosis [63]. Hence, it is still debated whether higher or lower SOD2 protein activity should be seen as a definite risk factor.

Glutathione peroxidase-1 is considered a gatekeeper able to stop detrimental damage caused by H_2_O_2_ produced by higher SOD2 activity [64]. In different stages of carcinogenesis, regulation of GPX1 levels is essential [65]. Many authors advocate SNP rs1050450 in the *GPX1* gene to contribute to susceptibility to various cancers [36, 66]. Namely, meta-analysis investigating the effect of this polymorphism revealed that variant genotypes (*Pro/Leu* and *Leu/Leu*) were associated with increased risk for lung cancer, bladder cancer, prostate cancer, head and neck cancer, and brain cancer [21, 67, 68]. However, Nikic et al. found no impact of *GPX1* polymorphism on overall survival in patients with metastatic urothelial bladder cancer [69]. Our results did not reveal increased risk for carriers of *Pro/Leu* and *Leu/Leu*; on the contrary, risk was reduced among these subjects. Follow-up analysis revealed that these variant allele carriers had shorter cumulative survival, but this was not statistically significant. This is not the first time to encounter that the Leu allele is associated with protection. Considering the fact that the variant GPX1 exhibits lower enzyme activity, the explanation of such phenomenon in ccRCC is challenging. However, as recently suggested, the roles of hydrogen peroxide in signal transduction and regulation of genes involved in longevity might have priority when compared to its potential to cause oxidative damage [70]. Further studies are needed to elucidate the mechanisms by which alteration in H_2_O_2_ reduction is associated with better survival and lower susceptibility to clear cell renal cell carcinoma.

Just recently, when expression of GPX1 protein was evaluated in RCC, high GPX1 level was in a positive correlation with tumor stage, distant metastasis, lymphatic metastasis, and shorter overall survival [24]. These contradictory results on the influence of *GPX1* polymorphism on both enzyme synthesis and activity should be further examined and revealed.

This study has several limitations that need to be addressed. The case-control study design and therefore selection bias, as well as the recall bias, regarding the recognized risk factors for ccRCC development might have influenced the results. Also, the control group was relatively small and comprised of hospital-based patients. Furthermore, the possible effect of ethnicity could not be evaluated as the study group consisted of Caucasians only.

## 5. Conclusions

Some important novel aspects regarding the role of SNPs in genes encoding the transcriptional factor Nrf2, mitochondrial SOD2, and GPX1 and *GSTP1ABCD* haplotype in pathophysiology of ccRCC are provided in this study. Namely, increased ccRCC susceptibility was observed among carriers of individual variant genotypes of both *SOD2* rs4880 and *GSTP1* rs1695 polymorphisms, as well as in combination with *Nrf2* rs6721961 genetic polymorphism. Furthermore, *GSTP1ABCD* haplotype analysis revealed significant risk of ccRCC development in carriers of the *GSTP1C* haplotype consisting of variant forms of both GSTP1 polymorphisms comprising this haplotype. Our study also provides evidence in favor of hypothesis that certain GST variant genotypes represent not only significant genetic risk factors for ccRCC development but also a significant prognostic factor. In this line, GSTP1 variant forms seem to affect the overall survival in patients with ccRCC and the proposed molecular mechanism underlying the role of GSTP1 forms in RCC progression might be the presence of GSTP1 : JNK1/2 protein : protein interactions.

## Figures and Tables

**Figure 1:** Kaplan-Meier survival curves for overall mortality according to (a) *Nrf2* polymorphism, (b) *GSTP1* polymorphisms rs1695 and rs1138272 in combination (*GSTP1*∗*reference* genotype—(Ile/Ile) (Ala/Ala); *GSTP1*∗*variant*-type genotypes—(Ile/Val+Val/Val)(Ala/Ala), (Ile/Ile)(Ala/Val+Val/Val), and (Ile/Val+Val/Val)(Ala/Val+Val/Val)), (c) *SOD2* polymorphism, and (d) *GPX1* polymorphism.

**Figure 2:** Expression of GSTP1 (23 kDa) protein analyzed by immunoblot in a pool of nontumor kidney tissue samples, as well as in ccRCC tissue samples (G1-G3). G1: tumor grade I; G2: tumor grade II; G3: tumor grade III. Expression of *β*-actin (42 kDa) protein in a pool of nontumor kidney tissue samples, as well as in ccRCC tissue samples (G1-G3), is used as a normalization control.

**Figure 3:** Expression of JNK1/2 (44/56 kDa) protein in a pool of nontumor kidney tissue samples, as well as in ccRCC tissue samples (G1-G3). G1: tumor grade I; G2: tumor grade II; G3: tumor grade III. Expression of *β*-actin (42 kDa) protein in a pool of nontumor kidney tissue samples, as well as in ccRCC tissue samples (G1-G3), is used as a normalization control.

**Figure 4:** Expression of cleaved caspase-3 (19/17 kDa) protein in a pool of nontumor kidney tissue samples, as well as in ccRCC tissue samples (G1-G3) (^∗^*p* < 0.05). Expression of *β*-actin (42 kDa) protein in a pool of nontumor kidney tissue samples, as well as in ccRCC tissue samples (G1-G3), is used as a normalization control.

**Figure 5:** Cytosols obtained from ccRCC tissue homogenates were immunoprecipitated with an anti-GST3/GST pi antibody. The samples were subjected to SDS-PAGE on 10% gel, followed by incubation with the primary antibodies against GST3/GST pi and JNK1/2. G1: tumor grade I; G2: tumor grade II; G3: tumor grade III; IP: immunoprecipitation; WB: Western blot.

**Table 1:** Baseline characteristics of ccRCC patients and age- and gender-matched controls.

	ccRCC patients	Controls	OR (95% CI^a^)	*p*
Age (years)^b^	58.95 ± 11.65	60.44 ± 10.84	/	0.125
Gender, *n* (%)				
Female	73 (33)	138 (41)	1.00^c^	
Male	147 (67)	198 (59)	1.467 (0.756-2.847)^d^	0.258
Obesity, *n* (%)^e^				
BMI < 25	65 (36)	110 (35)	1.00^c^	
BMI > 25	115 (64)	204 (65)	0.866 (0.494-1.518)^f^	0.616
BMI (kg/m^2^)	26.61 ± 4.43	26.78 ± 4.08	/	0.677
Smoking, *n* (%)^e^				
Never	82 (44)	164 (49)	1.00^c^	
Ever^g^	106 (56)	171 (51)	1.289 (0.863-1.925)^h^	0.215
Pack-years^i^	31 (0.30-96.00)	30.00 (0.20-88.00)	/	0.131
Hypertension, *n* (%)^e^				
No	83 (45)	211 (65)	1.00^c^	
Yes	102 (55)	116 (35)	2.450 (1.375-4.435)^j^	0.002
Tumor grade, *n* (%)^k^				
Grade I, G1	28 (15)			
Grade II, G2	106 (55)			
Grade III, G3	49 (26)			
Grade IV, G4	8 (4)			
pT stage, *n* (%)^k^				
pT1	93 (45)			
pT2	23 (11)			
pT3	87 (42)			
pT4	5 (2)			

^a^CI: confidence interval; ^b^mean ± SD; ^c^reference group; ^d^OR: odds ratio adjusted for age, BMI (body mass index), pack-years, and hypertension; ^e^based on the data available; ^f^OR adjusted for age, gender, pack-years, and hypertension; ^g^minimum of a 60-day period any time prior to the study onset; ^h^OR adjusted for age, gender, BMI, and hypertension; ^i^median (Min–Max); ^j^OR adjusted for age, gender, BMI, and pack-years; ^k^data available on patients' tumor grade and pT stage, depending on the type of surgery and pathohistological diagnostics.

**Table 2:** *Nrf2*, *SOD2*, *GPX1*, and *GSTP1* genotypes in relation to the risk of ccRCC.

Genotypes	ccRCC patients, *n* (%)	Controls, *n* (%)	OR (95% CI)^a^	*p*
*Nrf2* (rs6721961)				
C/C^c^	166 (77)	241 (72)	1.00^b^	
C/A and A/A^d^	50 (23)	95 (28)	0.692 (0.370-1.295)	0.250
*SOD2* (rs4880)				
Ala/Ala^e^	45 (30)	111 (21)	1.00^b^	
Ala/Val and Val/Val^f^	175 (70)	225 (79)	4.521 (2.167-9.432)	<0.001
*GPX1* (rs1050450)				
Pro/Pro^g^	109 (49)	142 (42)	1.00^b^	
Pro/Leu and Leu/Leu^h^	113 (51)	194 (58)	0.567 (0.323-0.994)	0.048
*GSTP1* (rs1695)				
Ile/Ile^i^	55 (25)	159 (47)	1.00^b^	
Ile/Val+Val/Val^j^	168 (75)	177 (53)	3.714 (1.952-7.069)	<0.001
*GSTP1* (rs1138272)				
Ala/Ala^k^	197 (89)	297 (89)	1.00^b^	
Ala/Val+Val/Val^l^	25 (11)	39 (11)	0.712 (0.309-1.642)	0.426
*GSTP1* (rs1695 and rs1138272)				
(Ile/Ile) (Ala/Ala)^m^	54 (24)	144 (43)	1.00^b^	
(Ile/Ile) (Ala/Val+Val/Val)^n^	1 (1)	15 (4)	0.000 (NA^q^)	0.999
(Ile/Val+Val/Val) (Ala/Ala)^o^	143 (64)	153 (46)	3.250 (1.668-6.331)	0.001
(Ile/Val+Val/Val) (Ala/Val+Val/Val)^p^	24 (11)	24 (7)	2.719 (0.970-7.624)	0.057

^a^OR: odds ratio adjusted for age, gender, BMI, pack-years, and hypertension; CI: confidence interval; ^b^reference group; ^c^C/C: carriers of both referent alleles; ^d^C/A and A/A: carriers of at least one variant allele; ^e^Ala/Ala: carriers of both referent alleles; ^f^Ala/Val and Val/Val: carriers of at least one variant allele; ^g^Pro/Pro: carriers of both referent alleles; ^h^Pro/Leu and Leu/Leu: carriers of at least one variant allele; ^i^Ile/Ile: carriers of both referent alleles; ^j^Ile/Val and Val/Val: carriers of at least one variant allele; ^k^Ala/Ala: carriers of both referent alleles; ^l^Ala/Val and Val/Val: carriers of at least one variant allele; ^m^(Ile/Ile) (Ala/Ala): carriers of both referent alleles for rs1695 and rs1138272; ^n^(Ile/Ile) (Ala/Val+Val/Val): carriers of both referent alleles for rs1695 and at least one variant allele rs1138272; ^o^(Ile/Val+Val/Val) (Ala/Ala): carriers of at least one variant allele for rs1695 and both referent alleles for rs1138272; ^p^(Ile/Val+Val/Val) (Ala/Val+Val/Val): carriers of at least one variant allele for both rs1695 and rs1138272; ^q^NA: not applicable.

**Table 3:** Combined effect of *Nrf2*, *SOD2*, *GPX1*, and *GSTP1* genotypes in relation to the risk of ccRCC carriers of at least one variant allele.

Genotypes	*Nrf2* (rs6721961)		*SOD2* (rs4880)		*GSTP1* (rs1695)		*GSTP1* (rs1138272)	
	C/C^c^	C/A and A/A^d^	Ala/Ala^e^	Ala/Val and Val/Val^f^	Ile/Ile^i^	Ile/Val+Val/Val^j^	Ala/Ala^k^	Ala/Val+Val/Val^l^
*Nrf2* (rs6721961) C/C^c^								
OR (95% CI)^a^	—	—	—	—	1.00^b^	3.211 (1.513-6.814)	1.00^b^	1.067 (0.41-2.779)
*p*	—	—	—	—	—	0.002	—	0.894
*Nrf2* (rs6721961) C/A and A/A^d^								
OR (95% CI)^a^	—	—	—	—	0.385 (0.095-1.564)	2.731 (1.107-6.739)	0.835 (0.430-1.621)	0.162 (0.019-1.408)
*p*	—	—	—	—	0.182	0.029	0.594	0.099
*SOD2* (rs4880) Ala/Ala^e^								
OR (95% CI)^a^	1.00^b^	0.308 (0.059-1.599)	—	—	1.00^b^	4.796 (0.927-24.81)	1.00^b^	0.594 (0.064-5.504)
*p*	—	0.161	—	—	—	0.062	—	0.646
*SOD2* (rs4880) Ala/Val and Val/Val^f^								
OR (95% CI)^a^	3.234 (1.436-7.280)	2.918 (1.131-7.532)	—	—	5.875 (1.190-29.00)	19.724 (4.267-91.16)	4.374 (2.012-9.508)	3.290 (1.054-10.26)
*p*	0.005	0.027	—	—	0.030	<0.001	<0.001	0.040
*GPX1* (rs1050450) Pro/Pro^g^								
OR (95% CI)^a^	1.00^b^	0.423 (0.158-1.133)	1.00^b^	3.653 (1.148-11.63)	1.00^b^	5.476 (2.127-14.10)	1.00^b^	0.826 (0.238-2.868)
*p*	—	0.087	—	0.028	—	*<0.001*	—	0.763
*GPX1* (rs1050450) Pro/Leu and Leu/Leu^h^								
OR (95% CI)^a^	0.440 (0.223-0.868)	0.456 (0.188-1.057)	0.553 (0.144-2.120)	2.533 (0.793-8.094)	0.720 (0.239-2.165)	2.194 (0.912-5.287)	0.585 (0.322-1.063)	0.372 (0.115-1.199)
*p*	0.018	0.067	0.388	0.117	0.558	0.079	0.079	0.098

^a^OR: odds ratio adjusted for age, gender, BMI, pack-years, and hypertension; CI: confidence interval; ^b^reference group; ^c^C/C: carriers of both referent alleles; ^d^C/A and A/A: carriers of both referent alleles; ^e^Ala/Ala: carriers of both referent alleles; ^f^Ala/Val and Val/Val: carriers of at least one variant allele; ^g^Pro/Pro: carriers of both referent alleles; ^h^Pro/Leu and Leu/Leu: carriers of at least one variant allele; ^i^Ile/Ile: carriers of both referent alleles; ^j^Ile/Val and Val/Val: carriers of at least one variant allele; ^k^Ala/Ala: carriers of both referent alleles; ^l^Ala/Val and Val/Val: carriers of at least one variant allele.

**Table 4:** Haplotype analysis of *GSTP1* rs1695 and rs1138272 polymorphisms in patients with ccRCC.

Genotype			Haplotype frequencies			
	rs1695	rs1138272	ccRCC patients, %	Controls, %	OR (95% CI)^a^	*p* value
*GSTP1A* ^d^	∗A	∗C	56	64	1.00^b^	
*GSTP1B* ^e^	∗G	∗C	38	30	1.50 (1.10–2.05)	0.012
*GSTP1C* ^f^	∗G	∗T	5	3	3.50 (1.49–8.22)	0.004
*GSTP1D* ^g^	∗A	∗T	1	3	0.00 (N/A^c^)	1.000
	Global haplotype association *p* value: <0.001					

^a^OR: odds ratio adjusted for age, gender, BMI, pack-years, and hypertension; CI: confidence interval; ^b^reference group; ^c^N/A: not applicable; ^d^*GSTP1A* genotype consisting of Ile105 and Ala114; ^e^*GSTP1B* genotype consisting of Val105 and Ala114; ^f^*GSTP1C* genotype consisting of Val105 and Val114; ^g^*GSTP1D* genotype consisting of Ile105 and Val114.

**Table 5:** *Nrf2*, *SOD2*, *GPX1*, and *GSTP1* genotype distribution among living and deceased ccRCC patients.

Genotype	Living patients, *n* (%)	Deceased patients, *n* (%)	*p* value
*Nrf2* (rs6721961)			
C/C^a^	99 (76)	59 (75)	
C/A and A/A^b^	31 (24)	19 (25)	0.530
*SOD2* (rs4880)			
Ala/Ala^c^	31 (24)	12 (15)	
Ala/Val and Val/Val^d^	101 (76)	68 (85)	0.093
*GPX1* (rs1050450)			
Pro/Pro^e^	57 (43)	46 (57)	
Pro/Leu and Leu/Leu^f^	77 (57)	34 (43)	0.024
*GSTP1* (rs1695 and rs1138272)			
(Ile/Ile) (Ala/Ala)^g^	41 (31)	12 (15)	
(Ala/Ala)(Pro/Leu+Leu/Leu) (Ala/Val+Val/Val)(Pro/Pro) (Ala/Val+Val/Val)(Pro/Leu+Leu/Leu)^h^	93 (69)	68 (85)	0.007

^a^C/C: carriers of both referent alleles; ^b^C/A and A/A: carriers of at least one variant allele; ^c^Ala/Ala: carriers of both referent alleles; ^d^Ala/Val and Val/Val: carriers of at least one variant allele; ^e^Pro/Pro: carriers of both referent alleles; ^f^ Pro/Leu and Leu/Leu: carriers of at least one variant allele; ^g^(Ile/Ile) (Ala/Ala): carriers of both referent alleles for rs1695 and rs1138272; ^h^carriers of at least one variant allele for either rs1695 or rs1138272.

**Table 6:** *Nrf2*, *SOD2*, *GPX1*, and *GSTP1* polymorphisms as predictors for overall mortality in patients with ccRCC.

Model 1^a^		Model 2^b^	
HR (95% CI)	*p* value	HR (95% CI)	*p* value
Risk for overall mortality comparing *Nrf2-variant*^c^ genotype to *Nrf2-reference*^d^-type genotype carriers			
1.030 (0.579–1.833)	0.919	1.104 (0.456–2.674)	0.826
Risk for overall mortality comparing *SOD2-variant*^e^ genotype to *SOD2-reference*^f^-type genotype carriers			
1.290 (0.676–2.461)	0.440	1.687 (0.494–5.755)	0.404
Risk for overall mortality comparing *GPX1-variant*^g^ genotype to *GPX1-reference*^h^-type genotype carriers			
0.737 (0.462–1.177)	0.201	1.388 (0.654–2.946)	0.393
Risk for overall mortality comparing *GSTP1-variant*^i^ genotype to *GSTP1-reference*^j^-type genotype carriers			
1.627 (0.664–3.986)	0.287	3.897 (0.681–22.304)	0.126

^a^Model 1 adjusted for age and gender; ^b^model 2 adjusted for the covariates from model 1 and recognized risk factors for ccRCC development (pack-years, BMI, and hypertension); ^c^*Nrf2-variant*-type genotype—C/A+A/A; ^d^*Nrf2-reference* genotype—C/C; ^e^*SOD2* variant-type genotype—Ala/Val+Val/Val; ^f^*SOD2* reference genotype—Ala/Ala; ^g^*GPX1-variant*-type genotype—Pro/Leu+Leu/Leu; ^h^*GPX1-reference* genotype—Pro/Pro; ^i^*GSTP1-variant*-type genotype—combination of genotypes of rs1695 and rs1138272 SNPs (Ile/Val+Val/Val) (Ala/Val+Val/Val); ^j^*GSTP1-reference* genotype—combination of reference genotypes of both rs1695 and rs1138272 (Ile/Ile) (Ala/Ala); HR: hazard ratio; CI: confidence interval.

## Data Availability

The data that support the findings of this study are available from the corresponding author (MPE) upon reasonable request.

## References

[1] Ursini F., Maiorino M., Forman H. J. (2016). Redox homeostasis: the golden mean of healthy living. *Redox Biology*.

[2] Mena S., Ortega A., Estrela J. M. (2009). Oxidative stress in environmental-induced carcinogenesis. *Mutation Research/Genetic Toxicology and Environmental Mutagenesis*.

[3] Pljesa-Ercegovac M., Savic-Radojevic A., Coric V., Radic T., Simic T. (2020). Glutathione transferase genotypes may serve as determinants of risk and prognosis in renal cell carcinoma. *BioFactors*.

[4] Ljungberg B., Albiges L., Abu-Ghanem Y. (2019). European Association of Urology guidelines on renal cell carcinoma: the 2019 update. *European Urology*.

[5] Protzel C., Maruschke M., Hakenberg O. W. (2012). Epidemiology, aetiology, and pathogenesis of renal cell carcinoma. *European Urology Supplements*.

[6] Chen F., Zhang Y., Şenbabaoğlu Y. (2016). Multilevel genomics-based taxonomy of renal cell carcinoma. *Cell Reports*.

[7] Pandey N., Lanke V., Vinod P. K. (2020). Network-based metabolic characterization of renal cell carcinoma. *Scientific Reports*.

[8] Fabrizio F. P., Costantini M., Copetti M. (2016). Keap1/Nrf2 pathway in kidney cancer: frequent methylation of Keap1 gene promoter in clear renal cell carcinoma. *Oncotarget*.

[9] Basak P., Sadhukhan P., Sarkar P., Sil P. C. (2017). Perspectives of the Nrf-2 signaling pathway in cancer progression and therapy. *Toxicology Reports*.

[10] Chartoumpekis D. V., Wakabayashi N., Kensler T. W. (2015). Keap1/Nrf2 pathway in the frontiers of cancer and non-cancer cell metabolism. *Biochemical Society Transactions*.

[11] Krajka-Kuźniak V., Paluszczak J., Baer-Dubowska W. (2017). The Nrf2-ARE signaling pathway: an update on its regulation and possible role in cancer prevention and treatment. *Pharmacology Reports*.

[12] Sporn M. B., Liby K. T. (2012). NRF2 and cancer: the good, the bad and the importance of context. *Nature Reviews. Cancer*.

[13] Cho H. Y., Marzec J., Kleeberger S. R. (2015). Functional polymorphisms in Nrf2: implications for human disease. *Free Radical Biology & Medicine*.

[14] Bartolini D., Galli F. (2016). The functional interactome of GSTP: a regulatory biomolecular network at the interface with the Nrf2 adaption response to oxidative stress. *Journal of Chromatography, B: Analytical Technologies in the Biomedical and Life Sciences*.

[15] Vasieva O. (2011). The many faces of glutathione transferase pi. *Current Molecular Medicine*.

[16] Coric V. M., Simic T. P., Pekmezovic T. D. (2017). GSTM1 genotype is an independent prognostic factor in clear cell renal cell carcinoma. *Urologic Oncology: Seminars and Original Investigations*.

[17] Board P. G., Menon D. (2013). Glutathione transferases, regulators of cellular metabolism and physiology. *Biochimica et Biophysica Acta (BBA) - General Subjects*.

[18] Bartolini D., Commodi J., Piroddi M. (2015). Glutathione S-transferase pi expression regulates the Nrf2-dependent response to hormetic diselenides. *Free Radical Biology & Medicine*.

[19] Pljesa-Ercegovac M., Savic-Radojevic A., Matic M. (2018). Glutathione transferases: potential targets to overcome chemoresistance in solid tumors. *International Journal of Molecular Sciences*.

[20] Hart P. C., Mao M., de Abreu A. L. P. (2015). MnSOD upregulation sustains the Warburg effect via mitochondrial ROS and AMPK-dependent signalling in cancer. *Nature Communications*.

[21] Cao M., Mu X., Jiang C., Yang G., Chen H., Xue W. (2014). Single-nucleotide polymorphisms of GPX1 and MnSOD and susceptibility to bladder cancer: a systematic review and meta-analysis. *Tumor Biology*.

[22] Wang Y., Branicky R., Noë A., Hekimi S. (2018). Superoxide dismutases: dual roles in controlling ROS damage and regulating ROS signaling. *The Journal of Cell Biology*.

[23] Miess H., Dankworth B., Gouw A. M. (2018). The glutathione redox system is essential to prevent ferroptosis caused by impaired lipid metabolism in clear cell renal cell carcinoma. *Oncogene*.

[24] Cheng Y., Xu T., Li S., Ruan H. (2019). GPX1, a biomarker for the diagnosis and prognosis of kidney cancer, promotes the progression of kidney cancer. *Aging (Albany NY)*.

[25] Lubos E., Loscalzo J., Handy D. E. (2011). Glutathione peroxidase-1 in health and disease: from molecular mechanisms to therapeutic opportunities. *Antioxidants & Redox Signaling*.

[26] Marzec J. M., Christie J. D., Reddy S. P. (2007). Functional polymorphisms in the transcription factor NRF2 in humans increase the risk of acute lung injury. *The FASEB Journal*.

[27] Reszka E., Jablonowski Z., Wieczorek E. (2014). Polymorphisms of NRF2 and NRF2 target genes in urinary bladder cancer patients. *Journal of Cancer Research and Clinical Oncology*.

[28] Ishikawa T. (2014). Genetic polymorphism in the NRF2 gene as a prognosis marker for cancer chemotherapy. *Frontiers in Genetics*.

[29] Okano Y., Nezu U., Enokida Y. (2013). SNP (-617C>A) in ARE-like loci of the NRF2 gene: a new biomarker for prognosis of lung adenocarcinoma in Japanese non-smoking women. *PLoS One*.

[30] Ding F., Li J. P., Zhang Y., Qi G. H., Song Z. C., Yu Y. H. (2019). Comprehensive analysis of the association between the Rs1138272 polymorphism of the GSTP1 gene and cancer susceptibility. *Frontiers in Physiology*.

[31] Yang X., Long S., Deng J., Deng T., Gong Z., Hao P. (2013). Glutathione S-transferase polymorphisms (GSTM1, GSTT1 and GSTP1) and their susceptibility to renal cell carcinoma: an evidence-based meta-analysis. *PLoS One*.

[32] Thévenin A. F., Zony C. L., Bahnson B. J., Colman R. F. (2011). GST pi modulates JNK activity through a direct interaction with JNK substrate, ATF2. *Protein Science*.

[33] Moyer A. M., Salavaggione O. E., Wu T.-Y. (2008). Glutathione S-transferase P1: gene sequence variation and functional genomic studies. *Cancer Research*.

[34] Li D., Dandara C., Parker M. I. (2010). The 341C/T polymorphism in the GSTP1 gene is associated with increased risk of oesophageal cancer. *BMC Genetics*.

[35] Atilgan D., Parlaktas B. S., Uluocak N. (2014). The relationship between ALA16VAL single gene polymorphism and renal cell carcinoma. *Advances in Urology*.

[36] Ratnasinghe D., Tangrea J. A., Andersen M. R. (2000). Glutathione peroxidase codon 198 polymorphism variant increases lung cancer risk. *Cancer Research*.

[37] Shimoyama Y., Mitsuda Y., Tsuruta Y., Hamajima N., Niwa T. (2014). Polymorphism of Nrf2, an antioxidative gene, is associated with blood pressure and cardiovascular mortality in hemodialysis patients. *International Journal of Medical Sciences*.

[38] Towbin H., Staehelin T., Gordon J. (1979). Electrophoretic transfer of proteins from polyacrylamide gels to nitrocellulose sheets: procedure and some applications. *Proceedings of the National Academy of Sciences of the United States of America*.

[39] Laemmli U. K. (1970). Cleavage of structural proteins during the assembly of the head of bacteriophage T4. *Nature*.

[40] Žuntar I., Kalanj-Bognar S., Topić E., Petlevski R., Štefanović M., Demarin V. (2004). The glutathione S-transferase polymorphisms in a control population and in Alzheimer’s disease patients. *Clinical Chemistry and Laboratory Medicine*.

[41] Foulkes A. S. (2008). *Applied Statistical Genetics with R*.

[42] Laborde E. (2010). Glutathione transferases as mediators of signaling pathways involved in cell proliferation and cell death. *Cell Death and Differentiation*.

[43] McIlwain C. C., Townsend D. M., Tew K. D. (2006). Glutathione _S_ -transferase polymorphisms: cancer incidence and therapy. *Oncogene*.

[44] Pajaud J., Kumar S., Rauch C., Morel F., Aninat C. (2012). Regulation of signal transduction by glutathione transferases. *International Journal of Hepatology*.

[45] Tew K. D., Townsend D. M. (2012). Glutathione-S-transferases as determinants of cell survival and death. *Antioxidants & Redox Signaling*.

[46] Ishii T., Itoh K., Takahashi S. (2000). Transcription factor Nrf2 coordinately regulates a group of oxidative stress-inducible genes in macrophages. *The Journal of Biological Chemistry*.

[47] Suzuki T., Shibata T., Takaya K. (2013). Regulatory nexus of synthesis and degradation deciphers cellular Nrf2 expression levels. *Molecular and Cellular Biology*.

[48] Hartikainen J. M., Tengström M., Kosma V. M., Kinnula V. L., Mannermaa A., Soini Y. (2012). Genetic polymorphisms and protein expression of NRF2 and sulfiredoxin predict survival outcomes in breast cancer. *Cancer Research*.

[49] Yuki H., Kamai T., Murakami S. (2018). Increased Nrf2 expression by renal cell carcinoma is associated with postoperative chronic kidney disease and an unfavorable prognosis. *Oncotarget*.

[50] Yamaguchi Y., Kamai T., Higashi S. (2019). Nrf2 gene mutation and single nucleotide polymorphism Rs6721961 of the Nrf2 promoter region in renal cell cancer. *BMC Cancer*.

[51] Holley S. I., Fryer A. A., Haycock J. W., Grubb S. E. W., Strange R. C., Hoban P. R. (2007). Differential effects of glutathione S-transferase pi (GSTP1) haplotypes on cell proliferation and apoptosis. *Carcinogenesis*.

[52] Jia C. Y., Liu Y. J., Cong X. L. (2014). Association of glutathione S-transferase M1, T1, and P1 polymorphisms with renal cell carcinoma: evidence from 11 studies. *Tumor Biology*.

[53] Coric V. M., Simic T. P., Pekmezovic T. D. (2016). Combined GSTM1-null, GSTT1-active, GSTA1 low-activity and GSTP1-variant genotype is associated with increased risk of clear cell renal cell carcinoma. *PLoS One*.

[54] Maniglia M. P., Russo A., Biselli-Chicote P. M. (2020). Glutathione S-transferase polymorphisms in head and neck squamous cell carcinoma treated with chemotherapy and/or radiotherapy. *Asian Pacific Journal of Cancer Prevention*.

[55] Pljesa-Ercegovac M., Savic-Radojevic A., Dragicevic D. (2011). Enhanced GSTP1 expression in transitional cell carcinoma of urinary bladder is associated with altered apoptotic pathways. *Urologic Oncology: Seminars and Original Investigations*.

[56] Tew K. D., Manevich Y., Grek C., Xiong Y., Uys J., Townsend D. M. (2011). The role of glutathione S-transferase P in signaling pathways and S-glutathionylation in cancer. *Free Radical Biology & Medicine*.

[57] Manevich Y., Hutchens S., Tew K. D., Townsend D. M. (2013). Allelic variants of glutathione S-transferase P1-1 differentially mediate the peroxidase function of peroxiredoxin VI and alter membrane lipid peroxidation. *Free Radical Biology & Medicine*.

[58] Wang J., Liu Q., Yuan S. (2017). Genetic predisposition to lung cancer: comprehensive literature integration, meta-analysis, and multiple evidence assessment of candidate-gene association studies. *Scientific Reports*.

[59] Ma X., Chen C., Xiong H. (2010). No association between SOD2 Val16Ala polymorphism and breast cancer susceptibility: a meta-analysis based on 9, 710 cases and 11, 041 controls. *Breast Cancer Research and Treatment*.

[60] Crawford A., Fassett R. G., Geraghty D. P. (2012). Relationships between single nucleotide polymorphisms of antioxidant enzymes and disease. *Gene*.

[61] Mikhak B., Hunter D. J., Spiegelman D. (2008). Manganese superoxide dismutase (MnSOD) gene polymorphism, interactions with carotenoid levels and prostate cancer risk. *Carcinogenesis*.

[62] Sutton A., Imbert A., Igoudjil A. (2005). The manganese superoxide dismutase Ala16Val dimorphism modulates both mitochondrial import and MRNA stability. *Pharmacogenetics and Genomics*.

[63] Dasgupta J., Subbaram S., Connor K. M. (2006). Manganese superoxide dismutase protects from TNF-*α*-induced apoptosis by increasing the steady-state production of H2O2. *Antioxidants & Redox Signaling*.

[64] Ekoue D. N., He C., Diamond A. M., Bonini M. G. (2017). Manganese superoxide dismutase and glutathione peroxidase-1 contribute to the rise and fall of mitochondrial reactive oxygen species which drive oncogenesis. *Biochimica et Biophysica Acta (BBA) - Bioenergetics*.

[65] Brigelius-Flohé R., Kipp A. (2009). Glutathione peroxidases in different stages of carcinogenesis. *Biochimica et Biophysica Acta (BBA) - General Subjects*.

[66] Hu Y. J., Diamond A. M. (2003). Role of glutathione peroxidase 1 in breast cancer: loss of heterozygosity and allelic differences in the response to selenium. *Cancer Research*.

[67] Chen J., Cao Q., Qin C. (2011). GPx-1 polymorphism (Rs1050450) contributes to tumor susceptibility: evidence from meta-analysis. *Journal of Cancer Research and Clinical Oncology*.

[68] Wang C., Zhang R., Chen N. (2017). Association between glutathione peroxidase-1 (GPX1) Rs1050450 polymorphisms and cancer risk. *International Journal of Clinical and Experimental Pathology*.

[69] Nikic P., Dragicevic D., Savic-Radojevic A. (2018). Association between GPX1 and SOD2 genetic polymorphisms and overall survival in patients with metastatic urothelial bladder cancer: a single-center study in Serbia. *Journal of B.U.ON.*.

[70] Dragicevic B., Suvakov S., Jerotic D. (2019). Association of SOD2 (Rs4880) and GPX1 (Rs1050450) gene polymorphisms with risk of Balkan endemic nephropathy and its related tumors. *Medicina*.

